# Lyme rashes disease classification using deep feature fusion technique

This article has been retracted.

**DOI:** 10.1111/srt.13519

**Published:** 2023-11-06

**Authors:** Ghulam Ali, Muhammad Anwar, Muhammad Nauman, Muhammad Faheem, Javed Rashid

**Affiliations:** ^1^ Department of Computer Science University of Okara Okara Pakistan; ^2^ Department of Information Sciences Division of Science and Technology University of Education Lahore Pakistan; ^3^ School of Technology and Innovations University of Vaasa Vaasa Finland; ^4^ Department of IT Services University of Okara Okara Pakistan; ^5^ MLC Lab Okara Pakistan

**Keywords:** artificial intelligence, convolutional neural network classification, erythema migrans, fusion technique, Lyme disease

## Abstract

Automatic classification of Lyme disease rashes on the skin helps clinicians and dermatologists’ probe and investigate Lyme skin rashes effectively. This paper proposes a new in‐depth features fusion system to classify Lyme disease rashes. The proposed method consists of two main steps. First, three different deep learning models, Densenet201, InceptionV3, and Exception, were trained independently to extract the deep features from the erythema migrans (EM) images. Second, a deep feature fusion mechanism (meta classifier) is developed to integrate the deep features before the final classification output layer. The meta classifier is a basic deep convolutional neural network trained on original images and features extracted from base level three deep learning models. In the feature fusion mechanism, the last three layers of base models are dropped out and connected to the meta classifier. The proposed deep feature fusion method significantly improved the classification process, where the classification accuracy was 98.97%, which is particularly impressive than the other state‐of‐the‐art models.

## 1 INTRODUCTION

Good skin can help you feel confident, look younger for longer, and even prevent diseases.^1^ The skin maintains body temperature and protects the organs from fungi, germs, allergies, and viruses.^2^ Numerous factors contribute to the prevalence of skin problems among many people.^3^ The most common forms of skin diseases include psoriasis, eczema, alopecia, and ringworm.^4^ Similarly, Lyme disease is an infection caused by the bacterium Borrelia burgdorferi, transmitted to humans through the bite of infected ticks.^5^, ^6^ One of the most common Lyme disease symptoms is a rash known as erythema migrans, which can appear at the tick bite site. The common symptoms of Lyme disease include cardiovascular problems, neurological disorders, musculoskeletal troubles, and skin disorders.^7^, ^8^ Globally, Lyme disease is increasing in prevalence, and rising temperatures may contribute. British Medical Journal Global Health reports that 14.5% of the world's population has been infected with Lyme disease.^9^

Lyme disease association reported that more than 80 countries had reported cases of Lyme disease.^10^ According to the Centers for Disease Control and Prevention (CDC), there are around 476 000 new cases of Lyme disease recorded in the United States (US) every year.^11^ Lyme borreliosis affected about 12 400 Europeans in 2021.^12^ The highest rates are in Central and Western Europe features from data. Over the past decades, the accuracy (34.5%) and Asia (19.0%), and the most vulnerable are men aged 50 and up living in rural areas.^13^ The CDC estimated that approximately 300 000 people get Lyme disease yearly in Columbia.^14^ Lyme disease incidence in the United Kingdom is expected to double between 2020 and 2031, compared to 2011 to 2020.^9^

Various methods have been developed to diagnose Lyme disease.^15^ Sometimes symptoms overlap with those of other diseases, making diagnosis even for a seasoned rheumatologist difficult. Laboratory tests, such as the Western blot test, are used to find antibodies for a conclusive diagnosis^16^ after detecting potentially infected ticks. Medicine specialists recommended inappropriate antibiotics or unusual therapy for Lyme disease that caused cholecystitis, catheter‐associated bloodstream infection, venous catheter clogs, and fatality.^17^ Even in a developed country like the USA, less than 300 rheumatologists make them a very scarce specialty.^18^ The manual identification of Lyme disease is a callous and tiring process for patients.^19^ In addition, the right diagnosis is rare and heavily dependent on the physician's skills,^20^ and this treatment requires a diagnosis to lessen mortality loss.^18^ The inability of medical personnel to analyze Lyme disease processes is due to a lack of diagnostic expertise and the absence of a professional, computer‐aided diagnosis.^21^ Therefore, we must concentrate on developing more advanced medical technologies and an autonomous system that can identify Lyme disease quickly, accurately, and with minimal possibility of error.

Deep learning is a machine learning type that involves using artificial neural networks with multiple processing layers,^22^ which can automatically learn and extract features from data. Over the past 2 decades, the accuracy of disease predictions has grown by 15% to 20% because of machine learning (ML) algorithms.^23^ In the context of erythema migrans rash classification, deep learning methods could be used to extract features from images of rashes and use those features to classify the rashes as either indicative of Lyme disease or not.^24^

Deep feature fusion^25^ is a method proposed for this purpose, which merges the features extracted by different deep learning models to boost classification accuracy.^26^ Theoretically, this method could produce a more accurate representation of rash photos for classification purposes. Selecting and merging features is what feature fusion is all about; it is about how to eliminate extraneous or unimportant features.^27^ If the distributions of two traits are the same or nearly identical, they are redundant. A low correlation between a feature and the classes makes it irrelevant. Fusion of the remaining features yields an improved feature set, which is then fed into a classifier to produce the final result. As a result, to improve our classifications' precision, we focus on fusing decisions and features. However, the results of this study show that deep feature fusion is useful for rash classification in cases of erythema migrans. The best feature fusion techniques and deep learning models for erythema rash categorization are identified. The primary results of this research are as follows:

1. To develop a new feature fusion method based on deep neural networks that can differentiate between patients with Lyme positive (LP) infection and those with other disorders Lyme negative (LN).
2. To enhance the Lyme disease rashes, add images of patients collected from the different hospitals in Lahore, Pakistan.
3. To develop and boost the proposed method's performance in terms of classification accuracy.

The organization of this paper is as follows:

The following section briefly introduces the related works.
Section 3 explains the materials and methods, and the architecture of the proposed approach.
Section 4 provides experimental results and discussion where the effectiveness of the proposed scheme is compared to the existing schemes.
Finally, section 5 concludes this paper by summarizing our results, significance, limitations, and open issues for potential future work.

## 2 RELATED WORK

A few studies have explored using deep learning to classify erythema migrans rashes associated with Lyme disease. They used a convolutional neural network (CNN) to classify erythema migrans rashes based on images of the rashes. Alzubi et al.^17^ used the ResNet model for automatic Lyme disease diagnosis with an accuracy of 95.7% on random images dataset. The authors found that the CNN achieved high accuracy in the classification task and that using deeper networks (i.e., networks with more layers) resulted in better performance. Burlina et al.^28^ applied the ResNet50 for detecting erythema migrans and other baffling skin conditions using a cross‐sectional dataset of images, obtaining 95% accuracy in recognizing erythema migrans. Kehoe et al.^29^ constructed a discriminant model for Lyme illness based on metabolomics data, which is employed in general and can be readily adapted to other LCMS or metabolomics data sets.

Koduru et al.^30^ used deep convolutional neural networks trained on erythema migrans image classification with 93% accuracy. Servellita et al.^31^ developed a diagnostic classifier with an accuracy of 95.2% for the gene expression‐based detection of early Lyme illness. They used the limma package for linear modeling. Burlina et al.^32^ used random images for the detection of different types of skin lesions and achieved 93% accuracy. Vendrow et al.^33^ used a Lyme disease dataset to test their feature selection methods. Again, the Support Vector Machines model was used, and its accuracy was 72%. Hossain et al.^34^ use expert opinion assessment to improve a deep learning‐based Lyme disease classifier with patient data.

Pfeifer et al.^28^ worked on roughly 6080 images to train the dataset and applied several architectures (ResNet34, ResNet50, VGG19, and DenseNet121). Finally, the model trained with the DenseNet121 architecture achieved an accuracy of 80.72%. It is now possible to calculate the expected incidence rate of Lyme disease using machine learning, thanks to software developed by Chumachenko et al.^35^. Akbarian et al.^36^ used the ImageNet dataset. They used a computer vision approach by combining CNN and improved the accuracy of the image dataset by almost 92% for ticks, rashes, and Lyme disease.

Another study utilized a combination of CNNs and recurrent neural networks (RNNs) for erythema migrans rash classification. The authors found that RNNs, which are particularly well‐suited for processing sequential data, improved the model's performance. Burlina et al.^37^ developed a dataset and detected erythema migrans with 94% accuracy using machine learning. Jacob et al.^38^ used self‐supervised learning algorithms for Lyme disease classification with progressive resizing and referred to a self‐created dataset. Another study used XResNet‐18 and XResNet34 models for identifying the rash‐causing infection and got an accuracy rate of 84%. Pandiaraj et al.^39^ present good ways to diagnose Lyme disease in its early stages and clinical treatment procedures to motivate young researchers to be innovative. Johnson et al.^40^ created antibiotics and alternative treatments for chronic Lyme disease. Vendrow et al.^41^ use ML to examine Lyme data. Researchers use machine learning models to determine which factors suggest how researchers and participants rate their antibiotic response. A more recent study proposed deep feature fusion for erythema migrans rash classification. Zhou et al.^42^ worked on Deep Features Fusion with Mutual Attention Transformer for Skin Lesion Diagnosis. Almuayqil et al.^43^ worked on early signs of skin diseases using 118 multi types feature fusion models on the ImageNet dataset. The authors used multiple CNNs to extract features from rash images and combined the features using various fusion techniques. Radtke et al.^44^ used clinical data, achieved a LASSO logistic regression model, and got an accuracy of 95.5%. Aucott et al.^45^ utilized the Diffusion‐Convolutional Neural Networks (DCNN) model proposed for this skin lesion classifier, which has been made available to the general public to transfer learning to other models of skin lesion classification, and got an accuracy of 93.04%.

In prior research, we found that using deep feature fusion improved the performance of the classification task compared to using a single CNN model. Overall, these studies suggest that deep learning methods, including the use of deep feature fusion, have the potential to be effective for erythema migrans rash classification in the context of Lyme disease diagnosis. Also, the evidence suggests that prior datasets were not legit and authenticated by any skin doctor. There is a need to increase classification accuracy. However, more research is needed to fully understand the optimal approaches for using deep learning in this context also, as shown related work summary in Table 1.

**TABLE 1:** Overview of related work.

Reference	Methodology	Disease	Dataset	Accuracy (%)
^3^	CNN	Skin disease	ISIC archive	84
^17^	ResNet	Lyme disease	Lyme disease	95.7
^28^	Resnet50	Erythema migrans	Cross‐sectional	87
^29^	DCNN	Lyme rashes	Skin disease	90
^30^	Linear modeling	Erythema migran	Self‐created	75
^46^	CNN	Skin disease	Mylime data	95
^47^	CNN	Lyme disease	Online images	90
^48^	RNA‐Sequencing	Lyme disease	Random images	94
^49^	GrowCut	Skin lesions	Medical images	80
^50^	DCNN	Skin cancer	Isic	29

Abbreviations: DCNN, Diffusion‐Convolutional Neural Networks; CNN, convolutional neural network.

## 3 MATERIALS AND METHODS

Having a relevant and accurate dataset for the task at hand is crucial to the success of deep learning methodologies. The subsequent dataset is used in this study.

### 3.1 Dataset

Regarding the proposed procedure, experiments were carried out using the dataset obtained from Kaggle, which can be accessed online, named Lyme disease rashes.^51^ This dataset contains images of the infected patient's skin worms. Initially, 400 photos displaying common Lyme disease symptoms were found in the Lyme rashes disease dataset. Of these, 200 showed Lyme‐positive symptoms, whereas 200 showed Lyme‐negative signs. Because this dataset has several issues (Image labeling, Enhancement, etc.), which we identified after previewing it, we added an extra 192 Lyme‐positive and 118 Lyme‐negative photos collected from skin doctors from different hospitals in Lahore, Pakistan, and both of them verified all of the images in the dataset as depicted in Table 2 and the Figure 1.

**TABLE 2:** Lyme disease rashes dataset summary.

Class labels	Samples
Lyme positive	392
Lyme negative	318
Total	700

**FIGURE 1:** (A) Lyme disease positive (B) Lyme disease negative.

### 3.2 Image preprocessing

Preprocessing is used on all Lyme disease input photos to achieve more uniformity in classification results and better features. Overfitting might have been avoided by training on a large‐scale image dataset, which was necessary for the CNN approach to rash detection. It is the initial version of the Lyme rash illness dataset, which includes high‐resolution versions of every photograph in the dataset. We adjust the dimensions of the dataset to 224 × 224 with the help of python code. The model's performance will drastically decrease, but the processing time will be cut in half.

### 3.3 Data augmentation

Various data augmentation strategies were applied to prevent over‐fitting and boost the variety of the dataset. Using a scale transformation, as the parameter value was set to (1/255), the resulting pixel values all fell inside the range of zero to one. The photographs required a specific rotation; therefore, the rotation transformation was applied to them, requiring 25 degrees to achieve the desired outcome. The parameter height shift range was given the value of 0.1 to reposition the training images vertically. The random zoom transformation was applied using a zoom range of 0.2; a value greater than 1.0 indicates that the photographs were magnified, and a number much less than 1.0 indicates that the images were shrunk in size. The snapshot was flipped horizontally with the command Flip. The brightness transformation was employed. Therefore, the zoom range was from 0.5 to 1.0, where 0.0 indicates no brightness and 1.0 indicates maximum possible intelligence. The channel values are randomly transformed during the channel shift by selecting a value randomly from the available range. Because of this, we used a channel shift range of 0.05 and settled on fill mode to get the closest possible reproduction of the source material, as shown in Table 3.

**TABLE 3:** Data augmentation methods.

Methods used	Setting
Scaling	0 to 1 range
Rotation	25°
Zoom	0.2
Horizontal flip	True
True shear	20°

### 3.4 Dataset splitting

Lyme disease rash data was partitioned into a training, validation, and test set. Although the model was developed with the help of the training dataset, it was checked for accuracy using the validation set. Once the model was trained, it was tested on unseen photos (test set). There were 2074 photos of LP utilized for training, 691 for validation, and 691 for testing on the Lyme disease rash dataset. The remaining 1717, 572, and 572 images were used for training, validation, and test set of LN class, respectively. Total dataset of Lyme disease rash consisted of 3791 images for training, 1263 images of each validation, and test set of all classes. Table 4 displays a summary of the subset dataset.

**TABLE 4:** Dataset summary.

Class labels	Training	Validation	Testing	Total
LP	2074	691	691	3456
LN	1717	572	572	2861
Total	3791	1263	1263	6317

Abbreviations: LN, Lyme negative; LP, Lyme positive.

### 3.5 The proposed methodology

The development of deep learning technologies has brought about a revolution in machine learning and digital image processing. The ability of images to develop consistently, discriminate, and functional semantic properties give deep learning methods their potency. When we talk about making a network “deep,” we mean it has several layers. Not only is deep learning excellent at recognizing facial expressions,^52^ but it has also shown promise in other areas, such as smart city planning,^53^ skin cancer diagnosis,^54^ and so forth. Convolutional neural networks are the method of choice when dealing with image‐based issues. A threshold‐based deep learning model was developed to aid in diagnosing Lyme disease using imaging techniques. The data was gathered in‐house and pre‐processed with an adaptive histogram equalizer to eliminate unwanted variations. The proposed CNN model employs numerous permutations of layering. First, we will train three deep learning pre‐trained models to obtain or extract features from the last pooling layer in a vector form to classify affected and non‐affected rashes images. These pre‐trained models are InceptionV3, DenseNet201, and Xception. Second, the features extracted by the CNN layers will be concatenated and used for retraining the feature fusion's final classification “predictions” layer. At the same time, the base model will remain frozen. The obtained in‐depth features concatenate them. This approach is called feature fusion.

### 3.6 The architecture of the proposed deep feature fusion model

Any pattern recognition system aims to develop a highly accurate classification model for a given problem, such as diagnosing Lyme disease based on a patient's rash. Three initial models will be trained using Lyme disease rash symptoms data. The feature is extracted from a fully connected (Dense) layer, the output of which is a 2048‐dimensional vector in InceptionV3. A vector of 1000 dimensions represents each image's projected class scores. Features will be retrieved from the final pooling layer in the Xception model. It includes 2048 unique 8 × 8 map designs. DenseNet201, the global average pooling GAP, uses this layer as its penultimate pooling layer before the final fully connected layer, eliminating all remaining channels in the feature maps to produce an output of 1 × 1xC. It was repeated thrice with different parameters based on the results from the other locations and periods. An additional stage of meta‐classifier fusion is implemented. In the next phase, a novel feature fusion model will combine the extracted feature with others. We found that our model outperformed the state‐of‐the‐art methods. When we start working on feature fusion, all our pre‐trained models will stop receiving new data. The network's results are highly competitive with those from more traditional approaches. It is common practice to apply multiple classification models for a given pattern recognition job, each based on a different theory or set of methods, and then choose the one with the best overall performance. However, it was demonstrated that even if one model has the highest accuracy, the collections of patterns mistakenly classified by the multiple classifiers would only sometimes overlap. For this reason, adopting an ensemble approach with many classifiers can improve performance.^55^ This is because each classifier brings its distinct understanding of the classified patterns. Deep feature fusion‐based learning uses several agreeing models, as depicted in Figure 2, rather than relying on a single model to make a call.

**FIGURE 2:** The flowchart of the proposed model deep feature fusion.

After applying a cutoff to the classifier output probabilities (estimates of the posterior probability of the class), the hard‐level combination maps these probabilities into class labels.^56^ The majority voting technique considers the input from all classifiers that comprise a given hard‐level combination. The majority vote determines which category will be chosen. Deep feature level fusion has great potential to improve classification performance^57^, ^58^ since it combines many feature sets produced from different feature extractors. When many perspectives (in‐depth features obtained from multiple CNNs) must be represented, feature‐level fusion often involves concatenating numerous normalized feature subsets into a single feature vector. Concerning the CNN‐based feature‐level fusion studies, the finetuning of these CNN models using the same target dataset (the Lyme rashes disease dataset in our study) consisting of concatenated feature vectors can provide supplementary information.^59^ It is true even if the various CNN models are based on different configurations (or architectures). Feature fusion's numerical expression shifts based on the technique employed. Concatenation is a common technique for feature fusion, in which features from several sources are joined to create a new feature vector. This procedure can be expressed mathematically as:

(1) $$F_{f}used=\left[F_{1};\;F_{2};\;\text{…};F_{n}\right]$$

*F_f_* used is the fused feature vector, and *F_1_, F_2_, …*, and *F_n_* are the individual feature vectors from the different sources. The semi‐colon (;) represents concatenation.

Another standard method for feature fusion is element‐wise addition or averaging. The mathematical expression for this method would be:

(2) $$F_{f}used=\left(F_{1}+F_{2}+\cdots +F_{n}\right)/n$$

*F_f_* used is the fused feature vector, and *F_1_, F_2_, …*, and *F_n_* are the individual feature vectors from the different sources. The plus (+) sign represents element‐wise addition, and the division by *n* represents averaging. A more complex method is feature fusion through a Neural Network, where the feature vectors are passed through a neural network that learns to combine them optimally. In this case, the mathematical expression would depend on the neural network's architecture but involve matrix multiplication, activation functions, and biases. It's important to note that the feature fusion process can also be performed using a combination of different methods, and the mathematical expression will depend on the specific implementation.

#### 3.6.1 The first base model: InceptionV3

Szegedy et al.^60^ proposed an InceptionV3 model that employs a three‐inception‐block architecture, all of which feature parallel convolutions. Modules like this help relieve the over‐fitting issue and improve the computational efficiency of deep architecture. Annually, researchers in the Lyme disease image recognition and classification compete using 1.4 million photos from 1000 object classes for the ImageNet Large Scale Visual Identification Challenge (ILSVRC).^61^ Krizhevsky et al.^62^ suggest the AlexNet model and report substantial improvements in object identification and classification in their research. The Top‐5 error rate in object recognition and variety is then reduced by developing several convolutional models. Figure 3 of InceptionV3 depicts the top 5 error rates of object identification findings based on ImageNet, with GoogleNet displaying the most outstanding recognition results (InceptionV3). The results show that improving recognition performance can be achieved by making the model layer deeper. Regarding object identification, the InceptionV3 model outperforms its predecessor, GoogleNet (InceptionV1). The InceptionV3 model comprises the improved Inception module, the standard convolutional block, and the classifier. The first convolutional Lyme disease component is used in the feature following extraction, as shown in Figure 3.

**FIGURE 3:** InceptionV3 architecture diagram.

Layer types that switch between convolutional and max‐pooling, in which there is a Network‐In‐Network,^63^ form the foundation upon which the improved Inception module was built. This technique performs multiscale convolutions in parallel and then combines the convolutional results from each branch. It has been found that the introduction of auxiliary classifiers improves the consistency of training results, accelerates the rate at which gradients converge, and alleviates over‐fitting and vanishing gradient issues. The use of additional classifiers allows for these advantages to be realized. To reduce the required number of feature channels and quicken the training process, InceptionV3 uses the 1 × 1 convolutional kernel.

Furthermore, the massive convolution is split into smaller convolutions, reducing the total computation cost and the number of parameters. Therefore, this model is often employed for the function of transfer learning. In conclusion, InceptionV3's superior support system.

#### 3.6.2 The second base model: DenseNet201

It is a technique known as feed‐forward; all the layers that make up a Dense Convolutional Network (DenseNet) are connected. The number of feature maps in DenseNet is relatively low (12 filters per layer), and the layer itself is relatively thin (12 filters per layer).^64^ The capabilities of DenseNet reduce the total number of parameters, and it has a minimal effect on the gradient problem, feature deployment, and feature reuse.^65^ However, the conventional L‐layer Convolutional Neural Network (CNN) has a relationship between its layers that is proportional to L(L+1), meaning that each layer builds upon the information from the previous layer. One such 201‐layer convolutional neural network is the DenseNet201. A network pre‐trained on over a million images is loaded from the ImageNet database. A thousand distinct types of objects, such as animals, plants, and technological gadgets, can be identified in a single image by the internet. As a result of this procedure, the network contains full feature representations for many different kinds of images. The most universally applicable input for the network is a 224‐by‐224‐pixel image. Each layer in the network is equipped with a filter‐based convolution, batch normalization (BN), and ReLU activation, as illustrated in Figure 4.

**FIGURE 4:** DenseNet201 architecture diagram.

It is possible to reduce the overfitting during training by initially passing through a batch normalization stage, a matrix representing each picture pixel. If the value is lower than that, ReLu will be triggered to change it; however, if the value is higher, it will not be changed and will continue to be used as is. At this stage, a ReLu‐activated matrix image is multiplied by a convolution matrix with a 3 × 3 filter. Another processed matrix will be the resultant value.

#### 3.6.3 The third base model: Xception

This research uses only depth‐separable convolution layers to create a neural network architecture for convolutional learning. Convolutional neural networks' feature maps are analyzed to see if they can be decoupled from cross‐channel and spatial correlations. The third base architecture is Xception (short for extreme Inception) since the idea behind it is more advanced than the one on which the Inception design was founded. The Xception design relies heavily on its network's 36 convolutional layers to glean valuable characteristics, as shown in Figure 5. After the input on top of a convolutional foundation, add a logistic regression layer. Additionally, fully‐connected layers can be included before the coating of logistic regression that will be the subject of the upcoming discussion of experimental evaluation. All modules containing the 36 convolutional layers are surrounded by linear residual connections, except for the first and end modules. The Xception architecture is a linear stack of depth‐separable convolution layers connected by residual links.

**FIGURE 5:** Xception architecture diagram.

### 3.7 Evaluation metrics

Precision, recall, and F1 scores were used to objectively evaluate the suggested model's performance in this study.

Accuracy refers to how well authentic and fake photos are identified. To calculate accuracy, one uses:

(3) $$\mathrm{ACC}\;=\;\left(\left(T\;P\;+\;T\;N\right)\right)/\left(T\;P\;+\;T\;N\;+\;F\;N\;+\;F\;P\right)\;\times \;100$$

Misclassified manipulated photos are false negatives (FN), whereas correctly classified ones are true positives (TP). The initial photos correctly identified are known as true negatives (TN), while those incorrectly labeled are known as false positives (FP). In the same way that it would be incorrect to label an altered image as genuine, it would also be incorrect to label a genuine image as altered.

An error model is one that consistently generates wrong results. It is how we keep track of the many times we were wrong.

(4) $$\mathrm{Error}\;=\;\left(\left(T\;P\;+\;F\;N\right)\right)/\left(T\;P\;+\;T\;N\;+\;F\;N\;+\;F\;P\right)\;\times \;100$$

The PPV measures how many times the model made correct positive predictions.

(5) $$P\;\mathrm{recision}\;=\;\left(T\;P\right)/\left(T\;P\;+\;F\;P\right)\;\times \;100$$

Recall, or sensitivity, is the fraction of true positives that the model captures.

(6) $$\mathrm{Recall}\;=\;\left(T\;P\right)/\left(T\;P\;+\;F\;N\right)\;\times \;100$$

The f1 score is a combination of the model's recall and its precision. The minimum is zero, and the highest is one. If it is the highest possible, that means the model is perfect.

(7) $$F\;1\;\mathrm{Score}\;=\;2\;\times \left(P\;\mathrm{recision}\;\times \;\mathrm{Recall}\right)/\left(P\;\mathrm{recision}\;+\;\mathrm{Recall}\right)\;\times \;100$$

### 3.8 Experimental setup

Using a Google Colab Pro account, we trained and tested the proposed and three baseline models. The next step was to train the model to automatically extract the deep feature from the last pooling layer of the underlying models. The proposed model and its three transfer learning basis models go through six iterations of training at a learning rate of 0.0001. The networks are trained using Adam (71), an adaptive first‐order gradient‐based optimization method. The batch size will be 16. If there is no improvement in the validation loss after five iterations, the learning rate is halved. Binary categorical cross entropy loss functions are used during training for all studies. When no other loss function is specified, cross‐entropy is used. Table 5 depicts the entirety of the experimental setup's configuration details.

**TABLE 5:** Experimental setup configuration details.

Configuration	Details
Base models	3 (InceptionV3, DesnseNet, Xception)
Platform used	Google Colab Pro
Epochs (all models)	6
Batch size	16
Learning rate	0.0001
Dropout factor	0.4
Optimizer	Adam
Loss function	Binary categorical cross entropy

## 4 RESULTS AND DISCUSSION

A publicly available dataset was used to evaluate the proposed methodology. In this section, we discuss the effectiveness of the proposed models and try to locate an alternative dataset for the same problem for comparative purposes. The enhancements made to the final model were determined after a series of studies. This section details the experiments and analyses that went into this study. Experiments were conducted to assess the effectiveness of the suggested model:

1. The proposed model's efficacy was evaluated on the Lyme rashes disease dataset.
2. Evaluate the suggested model against the best current alternatives.

### 4.1 The proposed deep fusion model performance analysis on the Lyme rashes disease dataset

The proposed model's accuracy and loss graphs on the Lyme rashes disease dataset during training and validation are shown in Figure 6. The proposed method's training accuracy begins at 97.54% and reaches 99.97% by the end of the final epoch. In comparison, the validation accuracy starts at 95.83% and reaches 99.04% by the end of the last epochs. From an initial 31.21% validation loss, it drops to a 3.84% loss by the era's end. Training losses are reduced from 38.14% to 2.2% throughout five epochs. The outcomes show that the proposed approach is highly effective, with extremely minimal training and validation loss and high levels of accuracy during both training and validation.

**FIGURE 6:** Accuracy, and loss graph of the proposed model.

The Lyme rashes disease dataset results show good performance across all categories. For further analysis, we compute the suggested technique's recall, precision, and F1 score on the test set, as depicted in Figure 7. Predictions of LP and LN statuses, respectively, are 98% and 100% precision using the suggested model (LN). The presented model attains 99.86% accuracy in the LP class, 97.9% in the LN class, and 98.97% overall accuracy, as shown in Table 6. It achieves 99% F1 scores across all classes and 100% recall across the LP, and 98% in the LN category.

**FIGURE 7:** The suggested method's classification accuracy, precision, recall, and f1 score.

**TABLE 6:** The proposed model's classification performance on the test set includes recall, precision, and f1 score.

	Lyme positive (LP) (%)	Lyme negative (LN) average (%)	Average (%)
Accuracy	97	99	98.97
Precision	97	99	–
Recall	100	98	–
F1 Score	99	99	–

Abbreviations: LN, Lyme negative; LP, Lyme positive.

The visual estimation of a model's classification accuracy using a confusion matrix is applied. The confusion matrix displays accurate predictions along the diagonal and inaccurate ones out to the side. A darker color indicates that the proposed model of the relevant class has a greater classification accuracy, whereas a lighter color indicates that misclassified samples are present. The confusion matrix on the test set is also used to evaluate the performance of the proposed base model. There are 1263 photos in the test set; 572 are in the LN category, and another 691 are in the LP category. A total of 560 LN photos are successfully identified by the proposed model. It means the proposed model is 97.92% accurate. The proposed model accurately classifies 690 images out of 691 total attempts, or 99.86% of the time. The proposed model achieves a false‐positive rate of only 1.03% for a 98.97% accuracy. The model achieves excellent results across all performance evaluation metrics when tested on LP and LN species, as shown in Figure 8.

**FIGURE 8:** The proposed model confusion matrix on test set.

On the Lyme rash disease dataset, the suggested technique produces high‐quality findings across all evaluation metrics.

### 4.2 Comparison analysis of the deep feature fusion technique with state‐of‐the‐art models

Here, the proposed model is compared to various top‐tier methods. In Table 7, we see the outcomes of a study that compares the most cutting‐edge algorithms for Lyme disease detection. Since a few previous researchers have only utilized the Lyme rashes disease dataset, we also compare it to other datasets to validate our approach. Table 7 shows that the deep stack learning model developed by Alzubi et al.^17^ has a 97% success rate when classifying various characteristics. Using a cross‐sectional dataset of photographs, Burlina et al.^37^ trained a ResNet50 to detect erythema migrans and other perplexing skin disorders; they achieved 95% accuracy in recognizing erythema migrans, but this only holds if the dataset is legitimate. For early Lyme disease identification based on gene expression, Servellita et al.^31^ created a diagnostic classifier with a 95.2% accuracy. Justin et al.^66^ trained a CNN to identify tick bites using a photo dataset collected via a mobile app. However, data on other skin conditions were included in the analysis. The proposed model considerably exceeds expectations, with an astonishing 98.97% accuracy, compared to the study reported in Table 7, which only attained 97%. Prior studies have yet to investigate these variables, either alone or in combination, and achieve a higher accuracy than our findings. As a result, we compare our deep fusion model to previous research. A suggestion for Lyme illness was created using the Deep Feature Fusion method, and its accuracy was measured at 98.97%. The results showed that the proposed Deep Feature Fusion technique model performed better than the cited study. It prevented a fair comparison of the study's findings to those of other, more reliable studies.^67^, ^68^, ^69^

**TABLE 7:** Assessment of the proposed strategy concerning state‐of‐the‐art paradigms.

Reference	Year	Method	Dataset	Accuracy (%)
^17^	2022	Stack ensemble	Lyme disease	97
^37^	2022	ResNet50	Cross‐sectional	95
^31^	2022	Linear modeling	Self‐created	95
^66^	2021	CNN	Public images	87
**The proposed method**		**Deep fusion**	**Lyme disease**	**98.97**

## 5 CONCLUSIONS AND FUTURE WORK

Lyme disease is a tick‐borne illness prevalent in many parts of the world. According to recent reports, the number of cases is increasing, highlighting the importance of adequate identification and classification methods. Current methods of diagnosis rely on a combination of clinical presentation, laboratory tests, and patient history. However, these methods can be time‐consuming and costly, and false‐negative results can occur. This research proposes a new technique for detecting Lyme disease based on deep learning algorithms. The proposed technique, called Deep Feature Fusion, utilizes a combination of three deep learning‐based models, namely DenseNet201, InceptionV3, and Xception. The models were trained and evaluated using a dataset of Lyme rashes disease images collected from patients with different disease subtypes. The proposed technique achieved an accuracy of 98.97%, significantly higher than other existing techniques. This study provides a promising avenue for the future detection and management of Lyme disease. Further research can be conducted to expand the use of the Deep Feature Fusion technique to identify other tick‐borne illnesses, such as Rocky Mountain spotted fever, and exclude Lyme disease when assessing the entire spectrum of skin diseases. The proposed technique can improve the accuracy and efficiency of Lyme disease detection, leading to earlier diagnosis and more effective treatment. This research presents a valuable contribution to Lyme disease detection and classification. The proposed technique can be integrated into clinical practice to improve the accuracy and efficiency of Lyme disease diagnosis, and it has the potential to impact the management of this growing global concern significantly.

## CONFLICT OF INTEREST STATEMENT

The authors have no conflict of interests.

## Data Availability

The data will be available upon request to the corresponding author.

## References

[1] Importance of Skin Health All Year Round. 2021. [Online]: https://www.rosemedicalgroups.org/blog/importance‐of‐skin‐health‐all‐year‐round#

[2] Aijaz SF , Khan SJ , Azim F , et al. Deep learning application for effective classification of different types of psoriasis. J Healthc Eng. 2022;2022:1‐12.10.1155/2022/7541583PMC878372335075392

[3] Voggu S , Rao KS . A survey on skin disease detection using deep learning techniques. J Algebr Stat. 2022;13(3):3916‐3920.

[4] Binol H , Plotner A , Sopkovich J , Kaffenberger B , Niazi MKK , Gurcan MN , Ros‐NET: a deep convolutional neural network for automatic identification of rosacea lesions. Skin Res Technol. 2020;26(3):413‐421.31849118 10.1111/srt.12817

[5] Melenotte C , Drancourt M , Gorvel JP . Post‐bacterial infection chronic fatigue syndrome is not a latent infection. Med Maladies Infect. 2019;49(2):140‐149.10.1016/j.medmal.2019.01.00630722945

[6] Patel R , Grogg KL , Edwards WD , Wright AJ , Schwenk NM . Death from inappropriate therapy for Lyme disease. Clin Infect Dis. 2000;31(4):1107‐1109.11049799 10.1086/318138

[7] Marzec NS , Nelson C , Waldron PR , et al. Serious bacterial infections acquired during treatment of patients given a diagnosis of chronic Lyme disease‐United States. Morb Mortal Wkly Rep. 2017;66(23):607.10.15585/mmwr.mm6623a3PMC565784128617768

[8] Filipescu SG , Butacu AI , Tiplica GS , Nastac DI . Deep‐learning approach in the study of skin lesions. Skin Res Technol. 2021;27(5):931‐939.33822405 10.1111/srt.13045

[9] Kluger J . Nearly 15% of People Worldwide Have Had Lyme Disease, 2022, [Online]: https://time.com/6187215/lyme‐disease‐more‐common/

[10] Arsenovic M . 32 Frightening Lyme Disease Statistics, 2022. [Online]: https://petpedia.co/lyme‐disease‐statistics/

[11] Bobe JR , Jutras BL , Horn EJ , et al. Recent progress in Lyme disease and remaining challenges. Front Med. 2021;1276.10.3389/fmed.2021.666554PMC841631334485323

[12] Sas A . Number of cases of Lyme borreliosis disease diagnosed in Poland from 2018 to 2021, 2023. [Online]: https://www.statista.com/statistics/1119311/number

[13] BMJ Health . More than 14% of world's population likely has (had) tick‐borne Lyme disease, 2023. [Online]: https://www.bmj.com/company/newsroom/more

[14] CDC . How many people get Lyme disease?, 2023. [Online]: https://www.cdc.gov/lyme/stats/humancases.html

[15] Liu S , Fan Y , Duan M , et al. AcneGrader: An ensemble pruning of the deep learning base models to grade acne. Skin Res Technol. 2022(5):677‐688.35639819 10.1111/srt.13166PMC9907630

[16] mayo clinic . Lyme disease. 2022. [Online]: https://www.mayoclinic.org/diseases‐conditions/lyme‐disease/diagnosis

[17] Alzubi A , Tiwari S , Walia K , et al. An efficient stacked deep transfer learning model for automated diagnosis of Lyme disease. Comput Intell Neurosci. 2022;2022:1‐9.10.1155/2022/2933015PMC890131535265109

[18] Levine B Why is it so hard to find a rheumatologist? 2019. [Online]: https://www.everydayhealth.com/rheumatoid‐arthritis/treatment/rheumatologist‐shortage/

[19] Bajwa MN , Muta K , Malik MI , et al. Computer‐aided diagnosis of skin diseases using deep neural networks. Appl Sci. 2020;10(7):2488.

[20] Bilal M , Ali G , Iqbal MW , et al. Auto‐Prep: efficient and robust automated data preprocessing pipeline. IEEE Access. 2022;10:107764‐107784.

[21] Gasmi S , Ogden NH , Leighton PA , et al. Practices of Lyme disease diagnosis and treatment by general practitioners in Quebec, 2008–2015. BMC Fam Pract. 2017;18:1‐8.28532428 10.1186/s12875-017-0636-yPMC5441092

[22] Kirubarajan A , Taher A , Shawn S , Masood S . Artificial intelligence in emergency medicine: a scoping review. J Amer Coll Emer Physicians Open. 2020;1(6):1691‐1702.10.1002/emp2.12277PMC777182533392578

[23] Anwar M , Abdullah AH , Altameem A , et al. Green communication for wireless body area networks: energy aware link efficient routing approach. Sensors. 2018;18(10):3237.30261628 10.3390/s18103237PMC6210318

[24] Brinker TJ , Hekler A , Enk AH , et al. Deep neural networks are superior to dermatologists in melanoma image classification. Eur J Cancer. 2019;119:11‐17.31401469 10.1016/j.ejca.2019.05.023

[25] Chen Y , Bhutta MS , Abubakar M , et al. Evaluation of machine learning models for smart grid parameters: performance analysis of ARIMA and Bi‐LSTM. Sustainability. 2023;15(11):8555.

[26] Khan AA , Madendran RK , Thirunavukkarasu U , Faheem M . D2PAM: epileptic seizures prediction using adversarial deep dual patch attention mechanism. CAAI Transact Intell Technol. 2023;8(3):755‐769.

[27] Mangai UG , Samanta S , Das S , Chowdhury PR . A survey of decision fusion and feature fusion strategies for pattern classification. IETE Technic Rev. 2010;27(4):293‐307.

[28] Anwar M , Masud F , Butt RA , et al. Traffic priority‐aware medical data dissemination scheme for IoT based WBASN healthcare applications. Comput Mater Contin. 2022;71(3):4443‐4456.

[29] Kehoe ER , Fitzgerald BL , Graham B , et al. Biomarker selection and a prospective metabolite‐based machine learning diagnostic for Lyme disease. Sci Rep. 2022;12(1):1478.35087163 10.1038/s41598-022-05451-0PMC8795431

[30] Koduru T , Zhang E . Using deep learning in Lyme disease diagnosis. J Stud Res. 2021;10(4).

[31] Servellita V , Bouquet J , Rebman A , et al. A diagnostic classifier for gene expression‐based identification of early Lyme disease. Commun Med. 2022;2(1):92.35879995 10.1038/s43856-022-00127-2PMC9306241

[32] Burlina P , Joshi N , Ng E , et al. Skin image analysis for erythema migrans detection and automated Lyme disease referral. Proceedings of OR 2.0 Context‐Aware Operating Theaters, Computer Assisted Robotic Endoscopy, Clinical Image‐Based Procedures, and Skin Image Analysis, October 2, 2018. Granada, Spain: Springer. 2018:244‐251.

[33] Vendrow J , Haddock J , Needell D , Johnson L . Feature selection from Lyme disease patient survey using machine learning. Algorithms. 2020;13(12):334.

[34] Hossain SI , de Herve JDG , Abrial D , et al. Expert opinion elicitation for assisting deep learning based Lyme disease classifier with patient data. Preprint posted online August 30, 2022. arXiv:2208.14384, 2022.

[35] Chumachenko D , Piletskiy P , Sukhorukova M , Chumachenko T . Predictive model of Lyme disease epidemic process using machine learning approach. Appl Sci. 2022;12(9):4282.

[36] Akbarian S , Nelder MP , Russell CB , et al. A computer vision approach to identifying ticks related to Lyme disease. IEEE J Transl Eng Health Med. 2021;10:1‐8.10.1109/JTEHM.2021.3137956PMC903782135492508

[37] Burlina PM , Joshi NJ , Mathew PA , et al. AI‐based detection of erythema migrans and disambiguation against other skin lesions. Comput Biol Med. 2020;125:103977.32949845 10.1016/j.compbiomed.2020.103977

[38] Jacob D , Nankar O , Gite S , Patil S , Kotecha K . Lyme disease detection using progressive resizing and self‐supervised learning algorithms lyme disease detection using progressive resizing and self‐supervised learning algorithms. SSRN, doi:10.2139/ssrn.4059738

[39] Pandiaraj S , Jose T , Velliangiri S . Investigation of smart methodologies in Lyme disease detection. Proceedings of the 2021 International Conference on Computer Communication and Informatics (ICCCI), April 21, 2021. Coimbatore, India: IEEE; 1‐5 2021.

[40] Iqbal MJ , Iqbal MW , Anwar M , et al. Brain tumor segmentation in multimodal MRI using U‐Net layered structure. Comput Mater Contin. 2022;74(3):5267‐5281.

[41] Vendrow J , Haddock J , Needell D , Johnson L . Feature selection on Lyme disease patient survey data. Preprint posted online August 24, 2020. arXiv:2009.09087, 2020.

[42] Zhou L , Luo Y . Deep features fusion with mutual attention transformer for skin lesion diagnosis. Proceedings of the 2021 IEEE International Conference on Image Processing (ICIP). Alaska, USA, 3797‐3801. IEEE; 2021.

[43] Almuayqil SN , El‐Ghany SA , Elmogy M . Computer‐Aided diagnosis for early signs of skin diseases using multi types feature fusion based on a hybrid deep learning model. Electronics. 2022;11(23):4009.

[44] Radtke FA , Ramadoss N , Garro A , et al. Serologic response to borrelia antigens varies with clinical phenotype in children and young adults with Lyme disease. J Clin Microbiol. 2021;59(11):e0134421.34379528 10.1128/JCM.01344-21PMC8525570

[45] Aucott J . Skin image analysis for erythema migrans detection and automated Lyme disease referral. Proceedings of the *OR 2.0* Context‐Aware Operating Theaters, Computer Assisted Robotic Endoscopy, Clinical Image‐Based Procedures, and Skin Image Analysis: First International Workshop, OR 2.0 2018, 5th International Workshop, CARE 2018, 7th International Workshop, CLIP 2018, Third International Workshop, ISIC 2018, Held in Conjunction with MICCAI 2018, June 14, 2018. Granada, Spain, 2018. Springer; 2018;11041:244.

[46] Joung HA , Ballard ZS , Wu J , et al. Point‐of‐care serodiagnostic test for early‐stage Lyme disease using a multiplexed paper‐based immunoassay and machine learning. ACS Nano. 2019;14(1):229‐240.31849225 10.1021/acsnano.9b08151

[47] Boligarla S , Laison EKE , Li JF , et al. Leveraging machine learning approaches for predicting potential Lyme disease cases and incidence rates in United States using twitter. Res Square. 2022;1‐16.10.1186/s12911-023-02315-zPMC1057802737845666

[48] Jutras BL , Bowman A , Brissette CA , et al. Ebfc (ybab) is a new type of bacterial nucleoid‐associated protein and a global regulator of gene expression in the Lyme disease spirochete. J Bacteriol. 2012;194(13):3395‐3406.22544270 10.1128/JB.00252-12PMC3434759

[49] Cuk E , Gams M , Moˇzek M , et al. Supervised visual system for recognition of erythema migrans, an early skin manifestation of Lyme borreliosis. Strojniˇski vestnik‐J Mech Eng. 2014;60(2):115‐123.

[50] Zafar M , Sharif MI , Sharif MI , et al. Skin lesion analysis and cancer detection based on machine/deep learning techniques: a comprehensive survey. Life. 2023;13(1):146.36676093 10.3390/life13010146PMC9864434

[51] Kaggle . 2023. [Online]: https://www.kaggle.com/datasets/sshikamaru/lyme‐disease‐rashes

[52] Rashid J , Shabbir Qaisar B , Faheem M , Akram A , Hamid M . Mouth and oral disease classification using InceptionResNetV2 method. Multimed Tools Appl. 2023:1‐19.

[53] Chu HH , Saeed MR , Rashid J , et al. Deep learning method to detect the road cracks and potholes for smart cities. Comput Mater Contin. 2023;75(1):1863‐1881.

[54] Rashid J , Ishfaq M , Ali G , et al. Skin cancer disease detection using transfer learning technique. Appl Sci. 2022;12(11):5714.

[55] Kittler J , Hatef M , Duin RP , Matas J , On combining classifiers. IEEE Trans Patt Anal Mach Intell. 1998;20(3):226‐239.

[56] Mohandes M , Deriche M Aliyu SO . Classifiers combination techniques: a comprehensive review. IEEE Access. 2018;6:19626‐19639.

[57] Saleem RM , Bashir RN , Faheem M , et al. Internet of things based weekly crop pest prediction by using deep neural network. IEEE Access. 2023;11:85900‐85913.

[58] Alarood AA , Faheem M , Al‐Khasawneh MA , Alzahrani AIA , Alshdadi AA . Secure medical image transmission using deep neural network in e‐health applications. Healthc Technol Lett. 2023;10(4):87‐98.37529409 10.1049/htl2.12049PMC10388229

[59] Zhou H , Ummenhofer B , Brox T . Deeptam.(2022); Deeptam: deep tracking and mapping. Proceedings of the European Conference on Computer Vision (ECCV), March 6, 2018. Munich, Germany: Springer; 2018:822‐838.

[60] Szegedy C , Vanhoucke V , Ioffe S , Shlens J , Wojna Z . Rethinking the inception architecture for computer vision. Proceedings of the IEEE Conference on Computer Vision and Pattern Recognition, September 24, 2016. IEEE; 2016:2818‐2826.

[61] Russakovsky O , Deng J , Su H , et al. Imagenet large scale visual recognition challenge. Int J Comput Vis. 2015;115:211‐252.

[62] Krizhevsky A , Sutskever I , Hinton GE . Imagenet classification with deep convolutional neural networks. Commun ACM. 2017;60(6):84‐90.

[63] Lin M , Chen Q , Yan S . Network in network. Preprint posted online December 16, 2020. arXiv:1312.4400, 2013

[64] Roslidar R , Saddami K , Arnia F , Syukri M , Munadi KA . A study of fine‐tuning CNN models based on thermal imaging for breast cancer classification. Proceedings of the 2019 IEEE International Conference on Cybernetics and Computational Intelligence (CyberneticsCom), October 21, 2019. Aceh, Indonesia: IEEE. 2019:77‐81.

[65] Ali G , Dastgir A , Iqbal MW , Anwar M , Faheem M . A hybrid convolutional neural network model for automatic diabetic retinopathy classification from fundus images. IEEE J Transl Eng Health Med. 2023;11:341‐350,

[66] Justen L , Carlsmith D , Paskewitz SM , Bartholomay LC , Bron GM . Identification of public submitted tick images: a neural network. Plos One. 2011;16(12):e0260622.10.1371/journal.pone.0260622PMC863893034855822

[67] Rashid J , Khan I , Ali G , et al. Real‐time multiple guava leaf disease detection from a single leaf using hybrid deep learning technique. CMC‐Comput Mater Contin. 2023;74(1):1235‐1257.

[68] Rashid J , Khan I , Ali G , et al. Multi‐level deep learning model for potato leaf disease recognition. Electronics. 2022;10(17):2064.

[69] Bock S , Weiß MA . Proof of local convergence for the Adam optimizer. Proceedings of the 2019 International Joint Conference on Neural Networks (IJCNN), September 30, 2019. Budapest, Hungary: IEEE. 2019:1‐8.

